The article "Effects of Nursing Care for the Treatment of Patients with Bladder Cancer: A Systematic Review and Meta-analysis" was retracted in 2023. Reasons: signs of a paper mill; compromised peer review; unreliable results or conclusions.

# Effects of Nursing Care for the Treatment of Patients with Bladder Cancer: A Systematic Review and Meta-analysis

**DOI:** 10.1155/2022/9554223

**Published:** 2022-09-25

**Authors:** Zhe Gao, Liang Fang, Peiyi Yin, Yan Deng, Mengting Pei, Tiantian Zhou

**Affiliations:** ^1^Department of Nursing, The Second Affiliated Hospital of Nanchang University, 330029, China; ^2^Department of Cardiothoracic Surgery, The Second Affiliated Hospital of Nanchang University, 330029, China

## Abstract

**Purpose:**

In this study, a systematic review and meta-analysis were used to examine the effectiveness of nursing care in the treatment of bladder cancer patients. The platforms of PubMed, Embase, Cochrane Library, and Web of Science were used to conduct a thorough literature search.

**Methods:**

The searching approach was used to find the fundamental characteristics of 5 studies. Sample size ranged from 52 to 131,852, and total sample size was 151,166. The study was looked up in PubMed, Embase, and Web of Science, with the most recent search being done in July 2022. Utilizing a standardized form, two independent reviewers gathered pertinent information from research that qualified as literature (17). Review Manager 5.3 used the data to examine the literature. Statistics were deemed significant at *p* < 0.05.

**Results:**

We discovered that more bladder cancer patients with T1+T2 tumor stages were receiving nursing care than those with T1+T2 tumor stages were receiving control care (mean difference =1.27, 95% CI: 1.20-1.35, *p* < 0.00001). The proportion of bladder cancer patients with T3+T4 tumor stage in the nursing care group was lower than the proportion of patients with T3+T4 tumor stage in the control group (mean difference = 1.07; 95% CI: 1.01-1.14; *p* < 0.00001). The difference between the number of bladder cancer patients receiving radiotherapy in the nursing care group and the control group was not statistically significant (mean difference = 1.07, 95% confidence interval [CI]: 0.99-1.16, *p* = 0.11). There were fewer patients with bladder cancer receiving chemotherapy in the nursing care group than that in the control group (mean difference = -0.02, 95% CI: -0.0-0.02, *p* < 0.00001). The incidence rate of patients with bladder cancer with major complications in nursing care group was lower than that of patients with bladder cancer with major complications in control group (mean difference = 0.41 95% CI: 0.18-0.93, *p* = 0.03). When compared to patients with bladder cancer who had serious complications in the control group, the hospital death rate for nursing care patients had a greater incidence of bladder cancer patients (mean difference = 4.64 95% CI: 4.46-4.82, *p* < 0.00001).

The article "Effects of Nursing Care for the Treatment of Patients with Bladder Cancer: A Systematic Review and Meta-analysis" was retracted in 2023. Reasons: signs of a paper mill; compromised peer review; unreliable results or conclusions.

**Conclusion:**

This study demonstrated that the effects of nursing care reduced the incidence rate of chemotherapy and the frequency of severe problems in bladder cancer patients.

## 1. Introduction

One of the most frequent malignant tumors of the urinary system, bladder cancer accounts for roughly 3.0 percent of new cases and 2.1 percent of cancer-related fatalities [1]. High incidence rate, prevalence, recurrence, and mortality of bladder cancer indicate that it is still an unsolved clinical and social problem [2]. Two-thirds of bladder cancer patients are nonmuscle invasive [2]. The 5-year survival rate for muscle invasive bladder cancer is about 60%, despite the fact that the current treatment has an excellent prognosis. After 5 years, roughly 40% of patients will develop muscle invasive bladder cancer [3].

The incidence rate and death of bladder cancer are complicated diseases impacted by a variety of variables [4]. The epidemiological characteristics of bladder cancer show obvious gender and age differences [5]. Men are more likely than women to develop bladder cancer, and as people age, they become more likely to develop the disease and die from it [6]. The incidence rate and death of bladder cancer will also be impacted by changes in population structure, various investigational techniques, and various reporting periods [7]. According to the aforementioned data, age, period, birth cohort, and other time factors may have an impact on the incidence rate and death of bladder cancer [8].

At present, surgical resection is the primary treatment for bladder cancer, but postoperative complications such as urinary tract infection, urinary leakage, incision infection, and intestinal obstruction will occur [4, 7, 8]. Some studies have shown that the incidence of early complications in patients with bladder cancer after total cystectomy is as high as 62%, leading to low quality of life and negative emotions such as anxiety and depression, which affect the physical and mental health of patients [5, 6, 9]. Continuous nursing can extend the nursing service to the community and families. It can not only effectively improve the self-care ability of patients with bladder cancer after operation and reduce the occurrence of complications, thus improving the quality of life of patients, but also improve the compliance of patients with medical treatment [10]. It can promote the disease recovery and daily life of patients with bladder cancer after discharge [11].

The popularization of bladder cancer-related knowledge is one of the main contents of bladder cancer continuing care services [12]. Some studies show that disease-related knowledge support can help cancer patients establish good confidence and improve their quality of life [13–15]. At present, there are various methods to popularize the disease-related knowledge of patients after bladder cancer surgery in China, including formulating health management manual, conducting knowledge lectures, and pushing articles on WeChat official account [16]. The formulation and distribution of the health management manual can effectively help patients master the knowledge related to bladder cancer, learn self-care skills, and improve the quality of life. The lectures on disease-related knowledge can not only popularize the related knowledge of patients and their families after bladder cancer surgery, but also answer the questions raised by patients, so as to improve the negative emotions such as anxiety and depression caused by the lack of disease knowledge [17]. The researchers used WeChat official account to push stoma knowledge, mental health knowledge, and abnormal situation treatment measures to patients and their families after bladder cancer surgery, which improved the patients' disease knowledge and self-care skills, and effectively reduced the complication rate of discharged patients [16]. Therefore, in the nursing process of discharged patients with bladder cancer, it is essential to publicize the disease-related knowledge [17].

The article "Effects of Nursing Care for the Treatment of Patients with Bladder Cancer: A Systematic Review and Meta-analysis" was retracted in 2023. Reasons: signs of a paper mill; compromised peer review; unreliable results or conclusions.

In the treatment for this kind of patients, total cystectomy and urinary diversion are radical schemes, including ileal replacement of bladder abdominal wall single stoma. The gold standard for treating bladder cancer includes in situ neobladders, ureteral abdominal wall double stomas, and other procedures [7]. Among them, operation time of bilateral abdominal stoma is shortened, and the postoperative complications are less. This operation is applicable to patients who are old, have basic diseases, and the body cannot tolerate long-term bladder replacement surgery [14]. However, the amount of care after surgery is doubled, and patients should take into account both sides of the stoma. It is inevitable that there will be omissions that will cause urine leakage and stimulate the skin, resulting in symptoms such as swelling and ulceration of the skin around the stoma. In addition, the postoperative urinary diversion, the loss of excretory function of normal physiological outlet, and the patients need to wear artificial bags for life result in the decline of quality of life [9]. Therefore, how to improve patients' self-care ability and reduce postoperative stoma complications, so as to improve their quality of life, has become a problem that clinical medical workers must solve. This study used a systematic review and meta-analysis to investigate the effectiveness of nursing home care in the management of individuals with bladder cancer.

The article "Effects of Nursing Care for the Treatment of Patients with Bladder Cancer: A Systematic Review and Meta-analysis" was retracted in 2023. Reasons: signs of a paper mill; compromised peer review; unreliable results or conclusions.

## 2. Materials and Methods

### 2.1. Literature Search

The study was looked up in PubMed, Embase, and Web of Science, with the most recent search being done in July 2022. The following are the MeSH terms and unrestricted words that were adopted: “Nursing care,” “Nursing,” “Care,” “Bladder cancer,” and “their combinations.” To locate other articles of interest, the reference lists of earlier pertinent evaluations were manually searched. The only language allowed for publishing was English.

### 2.2. Inclusion and Exclusion Criteria

The below inclusion criteria were employed to choose studies that qualified: When more than one publication from a patient cohort was found, the most comprehensive one was chosen. (I) The prognosis of bladder cancer was pathologically verified. The following things were excluded from consideration: (i) abstracts, reviews, case studies, or letters of comment; (ii) animal studies; (iii) publications that had already been published twice; and (iv) articles that had been written in a language other than English.

### 2.3. Data Extraction and Statistical Analysis

Utilizing a standardized form, two independent reviewers gathered pertinent information from research that qualified as literature (17). Review Manager 5.3 used the data to examine the literature (17). Using a Chi-square based *Q* test, where I2 denotes the degree of heterogeneity, heterogeneity across studies was investigated. Low heterogeneity was defined as *I*2 = 50% or pheterogeneity >0.1. For multiple comparisons, the data were analyzed via analysis of variance (ANOVA) with the Tukey-Kramer multiple comparisons test. Statistics were deemed significant at *p* < 0.05.

## 3. Results

### 3.1. Features of Included Studies and Characteristics of Included Studies

Through comprehensive literature searching, this paper was found utilizing a review and meta-analysis of the literature. The identification and evaluation of 198 literatures.  Table 1 displays the key characteristics of 5 investigations [18–22] from 2010 to 2021.  Figure 1 depicts the method used to choose the literature. The sample size ranged from 52 to 13 1,852, with a 151,166 overall sample size. The Cochrane Collaboration's technique for evaluating bias risk was used to assess the quality of the literature (Figures 2(a) and 2(b)). The several trials were double-blind, randomized, and used appropriate allocation concealment techniques (Figures 2(a) and 2(b)).

### 3.2. Effects of Nursing Care for Individuals with Bladder Cancer in Tumor Stage

The study examined how patients with bladder cancer's tumor stages were impacted by nursing care. We discovered that more bladder cancer patients with T1+T2 tumor stages were receiving nursing care than those with T1+T2 tumor stages receiving control category (mean difference =1.27, 95% CI: 1.20-1.35, *p* < 0.00001) (Figure 3(a)). T1 means that the tumor grows into the connective tissue beneath the endometrial layer. T2 means that the tumor invaded through the connective tissue into the muscle. While this was going on, fewer bladder cancer patients with T3+T4 tumor stages were receiving nursing care than those with T3+T4 tumor stages receiving control category (mean difference = 1.07, 95% CI: 1.01-1.14, *p* < 0.00001) (Figure 3(b)). These findings thus demonstrated that nursing care was primarily utilized in bladder cancer patients with T1+T2 tumor stages. The effectiveness of using T3+T4 tumor stage in bladder cancer patients to improve quality of life, however, remained uncertain.

The article "Effects of Nursing Care for the Treatment of Patients with Bladder Cancer: A Systematic Review and Meta-analysis" was retracted in 2023. Reasons: signs of a paper mill; compromised peer review; unreliable results or conclusions.

### 3.3. Effects of Nursing Care for Bladder Cancer Individuals along Treatment Factors

Next, we explored that the effects of nursing care affected on treatment factors of bladder cancer individuals. There were more individuals with bladder carcinoma receiving radiotherapy in the nursing care group than in the control group, but there was no statistically significant difference between the two groups of patients. (mean difference = 1.07, 95% CI: 0.99-1.16, *p* = 0.11) (Figure 4(a)). However, the quantity of individuals receiving chemotherapy for bladder cancer in the nursing care group was lower than the proportion of individuals receiving chemotherapy for bladder carcinoma in the control category (mean difference = -0.02, 95% CI: -0.02-0.02, *p* < 0.00001) (Figure 4(b)). These findings thus demonstrated that nursing care decreased the occurrence of bladder cancer patients receiving treatment. However, whether nursing care could increase the efficacy of chemotherapy in treatment with bladder cancer was unclear.

### 3.4. Effects of Nursing Care for Individuals with Bladder Carcinoma along Major Complications and Hospital Death

Lastly, this experiment explored that the effects of nursing care affected on complications and hospital demise of bladder carcinoma individuals. The occurrence rates for bladder carcinoma individuals with significant problems in the nursing care group were lower than those for bladder carcinoma individuals with significant complications in the control category (mean difference = 0.41 95% CI: 0.18-0.93, *p* = 0.03) (Figure 5(a)). These findings demonstrated that individuals with bladder malignancy experienced fewer significant problems because of nursing care. Nevertheless, the recurrence frequency of bladder cancer patients in the hospital nursing care group was higher than that of individuals with significant problems in the control category (mean difference = 4.64 95% CI: 4.46-4.82, *p* < 0.00001) (Figure 5(b)).

The article "Effects of Nursing Care for the Treatment of Patients with Bladder Cancer: A Systematic Review and Meta-analysis" was retracted in 2023. Reasons: signs of a paper mill; compromised peer review; unreliable results or conclusions.

### 3.5. Publication Bias

Publication bias “is a bias in the published literature, where the publication of research depends on the nature and direction of study results.” In Figure 6, funnel plots for a meta-analysis of serious complications and hospital deaths among bladder cancer patients are displayed. All of the analysis' funnel plots were symmetric, which excludes any publishing bias.

## 4. Discussion

Bladder cancer is one of the most prevalent malignant tumors of the urinary system and one of the cancers with the highest fatality rate (12). Bladder cancer had a standardized incidence rate of 6.69/100000 cases and a standardized death rate of 2.94/100000 cases worldwide in 2016. (13). In 2014, there were about 78100 new cases of bladder cancer in China, with a standardized incidence rate of 3.61/100000, about 32100 deaths, and a standardized mortality rate of 1.30/100000 [23]. Despite China has lower bladder cancer rates and fatality rates than the rest of the globe, it still shows an increasing trend in the past decade, and has become one of the important disease burdens in China [24]. Therefore, analyzing the changing trend of incidence rate, mortality, and disease burden of bladder cancer in China is conducive to the effective prevention and control of bladder cancer [25, 26]. According to our findings, 5 publications from 2010 to 20210 that covered 151166 individuals were encompassed in meta-analysis. The percentage of bladder cancer patients with T1+T2 tumor stages in the nursing care group was higher than the percentage of patients with T1+T2 tumor stages in the control category. The proportion of bladder tumor individuals with T3+T4 tumor stage in the nursing care group was lower than the proportion of individuals with T3+T4 tumor stage in the control category.

In China, the prevalence of bladder cancer is the highest among malignant tumors of the urinary system and is rising [13]. Radical cystectomy plus permanent urinary diversion is the main surgical method for the treatment of recurrent and multiple invasive bladder cancer [14]. Abdominal wall urinary diversion is a permanent urinary diversion that opens the urinary tract to the abdominal wall and discharges urine out of the body [14]. The operation has changed the patient's normal urination mode. After urinary diversion, the patient must wear a urine bag for life, which has seriously damaged the patient's physical image, resulting in greater postoperative psychological stress response, decreased self-esteem and self-efficacy, and then weakened confidence in life control and future life [17]. This reduces the quality of life of patients to a certain extent, increases their care needs, and produces dependence on nurses and caregivers. Nursing dependence is a kind of care relationship with professional characteristics. Its concept originates from Orem's theoretical research [16]. When individuals have self-care defects, nurses or caregivers need to provide compensatory help corresponding to their nursing needs. Studies have shown that patients' nursing dependence behavior is closely related to quality of life [27]. Excessive nursing dependence behavior will increase the risk of reducing the health status of patients and even threaten the lives of patients. Understanding the current state of affairs and the variables that affect nursing reliance in individuals with bladder carcinoma is crucial (21). According to the current study, there were fewer patients with bladder cancer receiving chemotherapy in the nursing care group than in the control group. These findings demonstrated that nursing care decreased the prevalence of bladder cancer patients receiving chemotherapy.

The article "Effects of Nursing Care for the Treatment of Patients with Bladder Cancer: A Systematic Review and Meta-analysis" was retracted in 2023. Reasons: signs of a paper mill; compromised peer review; unreliable results or conclusions.

These findings thus demonstrated that nursing care decreased the incidence rate of bladder cancer patients receiving treatment. However, whether nursing care could increase the efficacy of chemotherapy in treatment with bladder cancer was unclear.

After consulting the literature, the concept of the core nursing problems of elderly bladder cancer radical surgery was not retrieved [28]. According to the definition of “core nursing outcomes” by Iowa College of Nursing and previous research, the most prevalent nursing issues that can capture the essence of nursing care for elderly patients undergoing radical bladder tumor surgery are considered the study's key nursing issues [29, 30]. According to these studies, the incidence rate of bladder cancer patients who experienced serious complications was lower in the nursing care group than in the control category (mean difference = 0.41 95 percent CI: 0.18-0.93, *p* = 0.03). The incidence rate of bladder cancer patients in the hospital death of nursing care category was greater than the incidence rate of bladder cancer patients in the control group with substantial difficulties (mean difference = 4.64 95 percent CI: 4.46-4.82, *p* < 0.00001). These findings demonstrated that individuals with bladder malignancy experienced fewer significant problems because to nursing care.

The discharged patients after bladder cancer surgery suffer great pressure on their physiology and psychology due to large surgical trauma, changes in the original urination mode, and easy complications, which seriously affect the quality of life of the patients and their families [8, 31]. Therefore, bladder cancer patients have a great demand for continuous care services [17]. The research shows that the continuous nursing of patients after bladder cancer surgery has made initial development in China [16]. The implementation of continuous nursing can improve the degree of disease knowledge and self-care ability of discharged patients with bladder cancer, reduce the occurrence of complications, improve the quality of life of patients, and promote their health [32, 33]. However, there are still many problems in the continuous care of bladder cancer patients in China. First, the content of continuous care services is not standardized. There are many forms and contents of continuous care services for bladder cancer patients in China, but no effective continuous care services and systems for bladder cancer have been established. Also, there are great differences in the content of care services in different regions and hospitals. Second is the imperfect community service: The community health service centers in China mainly focus on general medicine, and lack of specialized personnel, which limits the coverage and coverage of health services and cannot meet the needs of nursing services for patients after bladder cancer surgery. Third, the continuous care of patients' caregivers is not highly concerned: cancer not only affects the quality of life of patients, but also has a certain impact on the quality of life of their caregivers. At present, the continuing care service for bladder cancer patients in China is mainly aimed at bladder cancer patients, but the degree of care for their caregivers is not high. Finally, insufficient resource allocation of stoma clinic: Opening a stoma clinic can provide stoma-related knowledge and comprehensive nursing services for patients undergoing stoma after bladder cancer surgery [18, 34, 35]. Although stoma clinic has been developed in China in recent years, the trained professionals can hardly meet the nursing needs of huge stoma patients [36].

The article "Effects of Nursing Care for the Treatment of Patients with Bladder Cancer: A Systematic Review and Meta-analysis" was retracted in 2023. Reasons: signs of a paper mill; compromised peer review; unreliable results or conclusions.

Our present study has some limitations. Firstly, five literatures were identified and evaluated in this study. Because there were so few studies included, it was difficult to draw conclusions about how nursing care and bladder cancer are related. The second is how nursing care affects individuals with bladder cancer. To validate our findings, we will need to design high-quality, large-scale studies with more diverse patient populations. Furthermore, considerable heterogeneity was found for a number of characteristics; however, we utilized a fixed-effect model to account for the heterogeneity, which also existed since the included studies were different.

## Figures and Tables

**Figure 1:** Flow chart of this study.

**Figure 2:** Risk of included studies. Risk of bias summary (a). Risk of bias graph (b).

**Figure 3:** Effects of nursing care for patients with bladder cancer in tumor stage. T1+T2 tumor stage of patients with bladder cancer (a). T3+T4 tumor stage of patients with bladder cancer (b).

**Figure 4:** Effects of nursing care for patients with bladder cancer with treatment factors. Treatment factors, radiotherapy (a). Treatment factors, chemotherapy (b).

**Figure 5:** Effects of nursing care for patients with bladder cancer with major complications and hospital death. Major complications (a) and hospital death (b).

**Figure 6:** Publication bias of this study. T1+T2 tumor stage of patients with bladder cancer (a); T3+T4 tumor stage of patients with bladder cancer (b); treatment factors, radiotherapy (c); treatment factors, chemotherapy (d); major complications (e); and hospital death (f).

**Table 1:** Basic characteristics of included studies.

Study year	Country	Ethnicity	Total Cases	Cases (E/C)
Ismaeel [18]	USA	North America	294	29/265
Hugar [19]	USA	North America	8,794	2,728/6,066
Han [20]	China	East Asia	131,852	13,224/118,628
Rabow [21]	USA	North America	52	30/22
Skolarus [22]	USA	North America	10,174	5,189/4,985

## Data Availability

The data used to support this study is available from the corresponding author upon request.
